# A Hemolysis Image Detection Method Based on GAN-CNN-ELM

**DOI:** 10.1155/2022/1558607

**Published:** 2022-02-22

**Authors:** Xiaonan Shi, Yong Deng, Yige Fang, Yajuan Chen, Ni Zeng, Limei Fu

**Affiliations:** College of Computer Science, Xi'an University of Science and Technology, Shanxi 710054, China

## Abstract

Since manual hemolysis test methods are given priority with practical experience and its cost is high, the characteristics of hemolysis images are studied. A hemolysis image detection method based on generative adversarial networks (GANs) and convolutional neural networks (CNNs) with extreme learning machine (ELM) is proposed. First, the image enhancement and data enhancement are performed on a sample set, and GAN is used to expand the sample data volume. Second, CNN is used to extract the feature vectors of the processed images and label eigenvectors with one-hot encoding. Third, the feature matrix is input to the map in the ELM network to minimize the error and obtain the optimal weight by training. Finally, the image to be detected is input to the trained model, and the image with the greatest probability is selected as the final category. Through model comparison experiments, the results show that the hemolysis image detection method based on the GAN-CNN-ELM model is better than GAN-CNN, GAN-ELM, GAN-ELM-L1, GAN-SVM, GAN-CNN-SVM, and CNN-ELM in accuracy and speed, and the accuracy rate is 98.91%.

## 1. Introduction

Hemolysis is the process by which the red blood cell membrane breaks down, and the hemoglobin in the cell is released into plasma, serum, and other intercellular substances. This abnormal expression can easily lead to many diseases. In particular, neonatal hemolysis has become one of the most important diseases affecting newborn health [1, 2]. In 2018, Zhang [3] analyzed 200 cases of neonatal jaundice. Neonatal hemolysis occurred in 61.61% of the 99 female infants. Among 101 baby boys, neonatal hemolysis accounted for 50.49%. Thus, it can be seen that the probability of jaundice caused by hemolysis of newborns is still relatively high. However, many patients become sicker and even lose their lives since hemolysis is not detected early enough [4].

In clinical hemolysis tests, the specimen character and quality judgment need to be visually measured and recorded by medical staff one by one, and the degree of hemolysis is easily affected by subjective factors. A Vitros 5600 biochemical immune analyzer is used to detect the hemolysis index, realizing automatic quantitative determination of the hemolysis degree [5] and avoiding errors and missing terms caused by manual operation. The concentration of NSE in neonatal hemolysis samples is calculated by the neuron-specific enolase (NSE) correction formula, which avoided repeating sample collection. It is particularly difficult to collect blood samples from newborns [6]. These methods rely on chemical instruments and the practical experience of medical personnel. The measurement of relevant data is complex and takes a long time.

In recent years, with the rapid development of deep learning technology, computer-aided detection technology has provided better results than traditional methods [7, 8]. In particular, medical image analysis provides medical personnel with more effective diagnostic and therapeutic procedures [9]. However, large-scale tagging data are difficult to obtain. Labeling medical data requires professional knowledge and invests considerable time and manpower. By training the existing data, generative adversarial networks (GANs) can automatically generate a large quantity of data to effectively solve this problem. For example, Qi et al. [10] generated a large number of diverse pulmonary nodule images through GAN, which saved time and cost. Convolutional neural networks (CNNs) also provide great help in medical image analysis. Huynh-the et al. [11] converted skeletal information into an image representation based on CNN. The experimental results with the highest accuracy were obtained on the most challenging datasets. Bueno et al. [12] achieved higher accuracy by using the sequential CNN segmentation-classification strategy. As a new training framework, the extreme learning machine (ELM) has been widely used in classification, identification, and diagnosis [13]. For example, Wang and Li [14] used ELM to classify pulse data, with an accuracy of 90.3%. Wang et al. [15] used the ELM method to quickly and accurately determine whether the human body has fallen. Cai et al. [16] verified the effectiveness and superiority of ELM in lithology identification through comparison.

To detect hemolysis images using computer-aided techniques instead of manual work and to improve the related algorithm, this paper proposes a hemolysis image detection method based on GAN-CNN-ELM. The prediction accuracy of this method is up to 98.91%, and the recognition accuracy and efficiency are better than GAN-CNN, GAN-ELM, GAN-ELM-L1, GAN-SVM, GAN-CNN-SVM, and CNN-ELM models. Furthermore, it realizes the efficient detection of hemolysis image and helps medical staff diagnose the condition in time and strives for more precious treatment time for patients.

This paper has three main contributions.

1. A large number of hemolysis images are generated by GAN to expand the dataset
2. The CNN algorithm is used to extract multilayer features from the preprocessed hemolysis experiment images
3. The ELM classifier is constructed to classify the eigenvalues and obtain more accurate prediction results

The paper is organized as follows.  Section 1 briefly describes the problems existing in hemolysis detection and the solution model. In Section 2, some specific methods adopted are introduced.  Section 3 gives the experimental process and results. Finally, in Section 4, several conclusions are presented, and the direction of our future work is mentioned.

## 2. Methodology

This paper presents an effective hemolysis image detection technique. The algorithm framework is shown in Figure 1. The main method includes three stages as follows:

- Image preprocessing
- CNN extraction features
- ELM classification

### 2.1. Image Preprocessing

The preprocessing of images mainly includes image segmentation and clipping, image enhancement, graphic transformation data enhancement, and generative adversarial network data enhancement. Image preprocessing is carried out with *X* images in *M* original image sets as the training atlas. *M*-*X* images represent the experimental atlas.

#### 2.1.1. Picture Initial Cropping and Labeling

*X* training pictures are segmented and cropped to obtain pictures of the hemolysis area in the test tube. Then, experts judged and labeled the hemolysis area and divided the images into three categories. The first category is insoluble, and the category number is 0, mainly based on the obvious precipitation in the test tube and obvious stratification. The second category is microsolubility, and the category number is 1. This is mainly based on the fact that the hemolysis solution in the test tube is partially precipitated, but the dissolution is relatively uniform in the upper layer, with obvious particles. The third category is the normal dissolution category, and the category number is 2, mainly based on the solution in the test tube dissolved evenly, excluding extreme cases (completely insoluble or clear water test tube); no larger particles or precipitation appeared. The results of the classification are shown in Figures 2 and 3.

#### 2.1.2. Image Enhancement

The collection of hemolysis images may be affected by uncontrollable factors such as light and photo angle, leading to the phenomenon of extremely concentrated grayscale of hemolysis images or unobvious feature areas [17, 18]. Therefore, image enhancement of the collected hemolysis image can cause different angle features and detail features of the image to appear, reduce the impact of irrelevant information, promote the model to extract more features of the image, and identify hemolysis from multiple features.

This algorithm mainly adopts histogram equalization [19] to enhance the image. For example, for a discrete grayscale image {*x*}, the number of occurrences of grayscale *i* is expressed as *n*_*i*_, and the probability of occurrence of pixels with grayscale *i* in the image is expressed as

(1) $$\begin{array}{c} p_{x}\left(i\right)=p\left(x=i\right)=\frac{n_{i}}{n},\;0\leq i<L, \end{array}$$

where *L* is all the grayscale numbers in the image, and the cumulative distribution function corresponding to *P*_*x*_ is defined as

(2) $$\begin{array}{c} \int {df}_{x}\left(i\right)=\overset{i}{\underset{j=0}{\sum }}p_{x}\left(j\right). \end{array}$$

In this paper, the probability distribution of the pixels of the original image on the grayscale level is changed by the method of histogram equilibrium to achieve the effect of image enhancement.

#### 2.1.3. Data Enhancement

Because of the unique characteristics of medical images, the position and angle of the subject image and other factors directly affect the judgment of the testing personnel. In CNN training, irregular images are likely to make model training unstable, resulting in the model not converging. Therefore, the data after image enhancement are enhanced to highlight the main information of the hemolytic image, standardize the dataset, and reduce the noise interference.

*(1) The Graphic Transformation*. The algorithm model adopts three methods of translation transformation, rotation transformation, and horizontal flipping to enhance the data [20–22].

*Image translation transformation*: assuming that there is a point *a* in the original image whose coordinates are (*x*, *y*), which is translated by *x*_0_ units along the *x*-axis and *y*_0_ units along the *y*-axis and the new coordinate is (*x*_1_, *y*_1_) = (*x* + *x*_0_, *y* + *y*_0_), its matrix expression is shown as

(3) $$\begin{array}{c} \left[\begin{array}{c} x_{1}\\ y_{1}\\ 1 \end{array}\right]=\left[\begin{array}{ccc} 1 & 0 & x_{0}\\ 0 & 1 & y_{0}\\ 0 & 0 & 1 \end{array}\right]•\left[\begin{array}{c} x\\ y\\ 1 \end{array}\right]. \end{array}$$

*Horizontal flip*: setting its original image width to width and height to height. The coordinates of one point in the original image is (*x*_0_, *y*_0_). After the horizontal mirror flip coordinates become (*x*_1_, *y*_1_) = (width − *x*_0_, *y*_0_), the matrix expression is represented as

(4) $$\begin{array}{c} \left[\begin{array}{c} x_{1}\\ y_{1}\\ 1 \end{array}\right]=\left[\begin{array}{ccc} -1 & 0 & \text{width}\\ 0 & 1 & 0\\ 0 & 0 & 1 \end{array}\right]•\left[\begin{array}{c} x_{0}\\ y_{0}\\ 1 \end{array}\right]. \end{array}$$

*Rotation transformation*: rotating the image clockwise around the origin by angle *θ*, then the coordinates of *x* after point (*x*, *y*) in the original image is changed to *x*cos*θ* − *y*sin*θ* and the coordinates of *y* is changed to *x*sin*θ* − *y*cos*θ*. The matrix expression is given as

(5) $$\begin{array}{c} \left[\begin{array}{c} a\left(x,y\right)\\ b\left(x,y\right)\\ 1 \end{array}\right]=\left[\begin{array}{ccc} \cos\theta & -\sin\theta & 0\\ \sin\theta & \cos\theta & 0\\ 0 & 0 & 1 \end{array}\right]•\left[\begin{array}{c} x\\ y\\ 1 \end{array}\right]. \end{array}$$

In this paper, the original image is first translated and transformed and then rotated at random angles. Finally, the image is randomly cropped to discard some irrelevant information in the image. Then, the data are expanded by means of horizontal inversion, and some error samples caused by excessive enhancement are removed.

*(2) Generative Adversarial Networks*. After the graph transformation, the unavailable samples are eliminated, resulting in a further reduction in the available training data. To solve the problem of insufficient training data, the existing data are trained by generating models to obtain a large amount of data to enhance the generalization ability of the network and improve the stability of the network and the universality of new samples.

GANs [23] are composed of two networks: a generator and a discriminator. The generator learns the distribution of real data as much as possible. The discriminator learns to judge whether the input data are from real data or generated data, and they play games and train against each other to finally reach the equilibrium state [24, 25].

Let the formula of sample *x* generated by a group of random noise *z* after the generator [17, 18] be as follows:

(6) $$\begin{array}{c} x^{\prime }=g\left(z,\theta_{g}\right), \end{array}$$

where*g* (*x*)is the final output after several convolution, pooling, and activation operations (see Equations (14) and (15), function with discriminator*D*_*f*_(*x*, *θ*_*g*_).

The output results of the real sample (*x*) and the generated sample (*x*′) after passing through the discriminator are shown in Equations (7) and (8).

(7) $$\begin{array}{c} x=D_{f}\left(x,\theta_{g}\right), \end{array}$$

(8) $$\begin{array}{c} x^{\prime }=D_{f}\left(x^{\prime },\theta_{g}\right). \end{array}$$

The discriminant result can be expressed as with the dichotomy result.

(9) $$\begin{array}{c} y=\left(\frac{D\left(x\right)}{D\left(x^{\prime }\right)}\right)=\left(\frac{D\left(x\right)}{D\left(G\left(z\right)\right)}\right), \end{array}$$

where *D*(*x*) represents the probability that *x* belongs to the real sample distribution, and the loss function [26, 27] is established. It is expressed as

(10) $$\begin{array}{c} \min_{G}\max_{D}V\left(G,D\right)=E_{x\sim P\text{data}}\left[\log D\left(x\right)\right]+E_{x\sim Pz}\left[\log\left(1-D\left(G\left(z\right)\right)\right)\right]. \end{array}$$

The GAN is optimized with a backpropagation algorithm.

When optimizing the generator, minimize *V*(*G*, *D*).Maximize *V*(*G*, *D*) when the discriminator is optimized. The gradient descent method can be used to optimize the solution so that the sample distribution generated by the generator is consistent with the actual sample.

### 2.2. CNN Feature Extraction

CNN is a biologically inspired neural network, which is composed of an input layer, several convolutional layers and pooling layers alternately, a fully connected layer, and an output layer. Among them, the convolution layer is used for convolution calculation, and the pooling layer is used for descending sampling. The main features of the image are extracted through these two layers. This algorithm uses the ResNet50 model [22] to extract features, as shown in Figure 4.

Assume that the input image matrix, the convolution kernel, and the feature map matrix are all in the form of a square. Here, the size of the input image matrix is *w*, the convolution kernel size is *k*, convolution kernels are *n*, convolution stride is *s*, zero-padding layer number is *p*, and the size of the *n* feature graphs generated by the convolution calculation is given as

(11) $$\begin{array}{c} W^{\prime }=\frac{w+2p-k}{s}+1. \end{array}$$

For an image after several layers of convolution, pooling operation, and the activation function, a number of feature graphs are obtained. Each feature graph is in matrix form, where *f*(∗) is the activation function. The Leaky ReLU function is selected in this paper.

(12) $$\begin{array}{c} y_{ij}=f\left(b+\overset{I}{\underset{i=0}{\sum }}\overset{w}{\underset{j=1}{\sum }}Wij\times Xij\right). \end{array}$$

After the convolution calculation of each pixel block in the image, the feature map matrix with the size of is obtained, as shown in the following equation:

(13) $$\begin{array}{c} \left[\begin{array}{ccc} y_{11} & \cdots & y_{1m}\\ \vdots & \ddots & \vdots \\ y_{n1} & \cdots & y_{nm} \end{array}\right]. \end{array}$$

The pooling operation is carried out. During the pooling process, the size of *k*∗*k* is selected as the pooling kernel. The calculation formulas of the two pooling modes are shown in Equations (14) and (15).

(14) $$\begin{array}{c} g\left(x\right)=\frac{\sum_{i=1}^{k*k}X_{i}}{k*k}, \end{array}$$

(15) $$\begin{array}{c} g\left(x\right)=\text{MA}{\text{X}}_{1\leq i\leq k}\left(X_{i}\right). \end{array}$$

After several operations, such as layer pooling, convolution, and activation, the last layer feature graph is expanded into the row vector, which is denoted as *Y*^*L*^, as the training data of ELM, where *φ* is the mapping function and V is the characteristic matrix.

(16) $$\begin{array}{c} Y^{L}=\phi \left(V\right). \end{array}$$

### 2.3. ELM Classification

By constructing the ResNet50 model, the pretrained model weight was loaded for feature extraction and preservation. The results of the last layer of the neural network are used for output. After each picture goes through the ResNet50 model, the feature vector L × 1 is extracted, where *L* is the feature number of each picture and *x* is the row vector, as shown in the following equation:

(17) $$\begin{array}{c} {\overset{⟶}{f}}_{i}=\left[x_{1},x_{2},\cdots x_{L}\right], \end{array}$$

corresponding to the one-hot code labeled3 × 1.

(18) $$\begin{array}{c} I_{i}=\left[{\text{I}}_{0},{\text{I}}_{1},{\text{I}}_{2}\right]. \end{array}$$

The N × L feature matrix is extracted from all image features to constitute the dataset for ELM [28] classification, where *N* represents the number of pictures and *L* represents the number of features.

(19) $$\begin{array}{c} F=\left[\begin{array}{c} f_{1}\\ f_{2}\\ \vdots \\ f_{N} \end{array}\right]=\left[\begin{array}{ccc} X_{11} & \cdots & X_{1L}\\ \vdots & \ddots & \vdots \\ X_{N1} & \cdots & X_{NL} \end{array}\right]. \end{array}$$

The ELM model is built as shown in Figure 5.

The implied nodes in the ELM network do not need to be adjusted through backpropagation (BP) but can be generated randomly based on a set of continuous probability distribution. The ELM contains two stages: a feature mapping stage and a learning stage. In this algorithm, the input data in the input layer is the image feature vector, and the output result of the *i*th node is shown in the following equation:

(20) $$\begin{array}{c} f\left(x_{i},w_{i},b_{i}\right)=x_{i}\cdot w_{i}+b_{i}. \end{array}$$

That is equivalent to mapping a *P*-dimensional vector to an *L*-dimensional vector.

(21) $$\begin{array}{c} h\left(x\right)=\left[g\left(x_{0},w_{0},b_{0}\right),\cdots ,g\left(x_{L},w_{L},b_{L}\right)\right], \end{array}$$

where *w*_*i*_ is the *i*th connection between the node of its input layer and the hidden layer, *b*_*i*_ is the bias, *g* is the activation function, and the sigmoid function is used here.

(22) $$\begin{array}{c} g\left(x_{i},w_{i},b_{i}\right)=\frac{1}{1+e^{-\left(x_{i}.w_{i}+b_{i}\right)}}. \end{array}$$

The number of nodes in the output layer is denoted as *M*, and the weight of the *i*th hidden layer node and the *j*th output layer node is *β*_*i*_. Then, the output (mapping) of node *j* is

(23) $$\begin{array}{c} f_{j}\left(x\right)=\overset{M}{\underset{i=1}{\sum }}\beta_{i}\cdot g\left(x,w,b\right)=h\left(x\right)\beta . \end{array}$$

In the learning stage, the characteristic matrix provided by the data of a given *m* training samples is denoted as *H*(*x*) = [*h*_1_(*x*), ⋯,*h*_*m*_(*x*)]^*T*^, which contains *m* mappings generated in the mapping phase. The objective function is represented as

(24) $$\begin{array}{c} \frac{1}{2}{\left\|H\beta -T\right\|}_{2}^{2}, \end{array}$$

where *β* is solved by the least squares.

(25) $$\begin{array}{c} \beta =\arg\min\left(\frac{1}{2}{\left\|H\beta -T\right\|}_{2}^{2}\right)=H*T, \end{array}$$

where *H*^∗^ is the generalized inverse moment of *H*.

To improve the generalization ability of the ELM model and avoid overfitting of the model, the *L*_1_ regular term [29] was added to the error function.

(26) $$\begin{array}{c} \frac{1}{2}{\left\|H\beta -T\right\|}_{2}^{2}+\alpha \left\|\beta \right\|. \end{array}$$

The solution of *β* is as follows:

(27) $$\begin{array}{c} \beta ={\left(H^{T}H+\alpha \cdot I\right)}^{-1}H^{T}. \end{array}$$

**I** is the unit matrix.

In summary, the steps of ELM training can be summarized as follows:

1. Initialize the hidden layer parameter (*w*_*i*_, *b*_*i*_) *i* = 1, ⋯, *L* according to the random continuous distribution
2. The output matrix ‖H‖ of the hidden layer is calculated according to Equations (15)–(18)
3. The weight matrix ‖*β*‖ is calculated according to Equation (22)

In the recognition stage, given a set of sample *X*, it first becomes *H*(*X*) after the mapping in the first stage; then, the category of the sample is given as

(28) $$\begin{array}{c} \text{label}\left(X\right)=\text{argmax}\left(H\left(X\right)\cdot \beta \right). \end{array}$$

The argmax function is the index that returns the largest value in the array; that is, the maximum probability category number is the prediction category.

## 3. Experiment

This experiment is carried out on a computer with 8 GB of 64-bit memory in Windows10, an i5-6200u CPU, and Python 3.6.

The dataset of this experiment is from the local medical institution, and the hemolytic blood samples are collected and labeled by professionals. The collection standard is the hemolysis index HI > 15. The original dataset for this experiment has 2250 hemolysis images used by medical laboratories with irregular resolution. Eighty percent (1800) of the original data are used as training data, and the remaining 20% (450) are used as final test data. The data distribution is shown in Table 1.

### 3.1. Dataset Processing

1. The image is segmented and cropped, and the random cropping resolution of the image is 128∗72. As a result, the training scale is expanded, and the clipped area is judged and classified. Histogram equalization is used to enhance the classified image, as shown in Figures 6 and 7

By redistributing the gray value of the original image, the gray value of the image is evenly distributed, so as to increase the contrast and enhance the details of the image. The gray histogram of Figure 6(a) is shown in Figure 8, and that of Figure 7(a) is shown in Figure 9.

(2) The quantity of data in the sample is initially expanded through graph transformation, and generative adversarial networks are used to conduct confrontation training on the data after graph transformation, and a large number of available training samples are generated, as shown in Figure 10. The number of training images generated in this experiment is 2350, and the original dataset is extended to 4600

### 3.2. Extraction of Image Features

Through image enhancement and data enhancement, the original data is utilized more efficiently. The generated samples are processed, and the unavailable samples are rejected. Then, feature extraction is conducted. In the process of feature extraction, three layers of feature maps are extracted for visual observation. The original insoluble hemolysis detection image is shown in Figure 11. After convolution and pooling operations at different scales, a number of feature maps are extracted from the original image to reflect the features of the original image from different angles, as shown in Figure 12.

### 3.3. Comparison of the ELM Training Effect

ELM has two parameters to determine in advance during training including the input to the model and the number of nodes in the hidden layer. Different parameters affect the training efficiency, fitting degree, and generalization effect of the model. The general principle is that the number of hidden nodes is less than the input dimension, and the number of features should not be too large.

In order to determine the appropriate size of the input layer and hidden layer, *K*-fold cross-validation is adopted in the analysis experiment to reduce overfitting and improve the generalization ability of the model, as shown in Figure 13. Experimental results show that 4-fold cross-validation has the highest accuracy, and 4-fold cross-validation is finally used to train GAN-ELM, GAN-ELM-L1, and GAN-CNN-ELM models. The initialization of hidden nodes is randomly generated based on a continuous probability distribution.

The training parameters are the number of selected features, and the influence of the hidden layer on accuracy is studied. The number of hidden nodes is selected as follows: 10, 100, 200, 400, 800, 1000, and 2000. Then, three models of GAN-ELM, GAN-ELM-L1, and GAN-CNN-ELM are trained separately under 4-fold cross-validation. The training results are shown in Figure 14.

As seen in the experimental results, when the number of hidden layer nodes *L* increased from 10 to 200, the accuracy is greatly affected and increased rapidly. From the stage of 400 to 800, the accuracy tended to be stable. After the 800th node, the model started to overfit, and the generalization ability is low. Therefore, the number of optimal hidden nodes is approximately 600, which has good performance in this experiment. The experimental results also show that the single ELM classifier is not effective. The accuracy is improved by adding a regularized ELM classifier, and the accuracy is greatly improved by the GAN-CNN-ELM classifier model.

After determining the optimal number of hidden nodes as 600, this paper adopts 4-fold cross-validation to verify the accuracy of each fold, as well as the accuracy of test set with and without cross-validation of the model. The experimental results are shown in Table 2. The experimental results indicate that the accuracy performance of the model in the final test set is improved after using 4-fold cross-validation.

### 3.4. Comparisons of Experimental Results

1. The traditional methods of hemolysis detection mainly include the Vitros 5600 biochemical immune analyzer to detect hemolysis indexes [5], the neuron-specific enolase (NSE) correction formula [6] and microcolumn gel detection card [30]. Because these experimental methods do not rely on human subjective judgment, it avoids the influence of human subjective factors and improves the accuracy of detection. At the same time, it does not rely on chemical instruments, saves chemical reagents, and is simple to operate. Computers operate much faster than physical and chemical analysis instruments. Therefore, it avoids the drawback of time-consuming measurement of relevant data and improves the detection efficiency to a large extent
2. This experiment compared seven different algorithms: GAN-CNN, GAN-ELM, GAN-ELM-L1, GAN-SVM, GAN-CNN-SVM, CNN-ELM, and GAN-CNN-ELM. The results show that the training model of the GAN-CNN-ELM classifier is adopted, since GAN greatly increased the sample data; compared with the CNN-ELM algorithm, the feature extraction time increased, but the accuracy improved. As the full connection layer in CNN network structure requires backpropagation to adjust parameters, ELM is a single hidden layer feedforward neural network, and the weight of the input layer and bias of hidden layer are randomly selected. ELM is used to replace the full connection layer for feature classification, which effectively reduces the computational complexity of the algorithm and improves the efficiency of model detection. The GAN-CNN-ELM model was compared with other models; the training time and accuracy are optimized. In Table 3, the accuracy is increased by at least 0.16%

Four models with relatively high accuracy are selected: GAN-CNN, GAN-CNN-SVM, CNN-ELM, and GAN-CNN-ELM. The remaining 20% of test data are into different models that are trained for prediction. The results are shown in Table 4.

Through the above experimental comparison, the results show that the GAN-CNN-ELM algorithm model is significantly better than the other three models in terms of recognition time and recognition accuracy. The recognition accuracy is increased by at least 2.58%.

## 4. Conclusion

This paper proposes a GAN-CNN-ELM algorithm model for hemolysis image detection, which uses image enhancement and graphic transformation to enhance image features and expand sample data. Then, we use the GAN to train the existing data to obtain a large quantity of data. The ResNet50 algorithm model is used to extract multilayer features of the pretreated hemolytic experimental atlas. The ELM classifier is constructed to classify the feature values to improve training time efficiency. For the test set, the accuracy of identification is as high as 98.91%. To achieve efficient identification of hemolytic images and accurately determine the hemolytic results.

In the future, multiscale convolution can be used to optimize the generalization degree of the system and the diversity of the recognition. An attempt will be made to improve the accuracy with CNN multiple feature fusion (MFF). The Res2Net framework will be used to extract multilayer features of the image to make the granularity finer and the feature scale more diverse, and the KELM algorithm will be studied to further improve the model training speed.

## Figures and Tables

**Figure 1:** Algorithm framework.

**Figure 2:** Image classification of the hemolysis area.

**Figure 3:** Classification of hemolysis images of different categories.

**Figure 4:** Schematic diagram of the ResNet50 algorithm model.

**Figure 5:** ELM model.

**Figure 6:** Original image.

**Figure 7:** Image enhancement process.

**Figure 8:** Gray histogram of Figure 6(a).

**Figure 9:** Gray histogram of Figure 7(a).

**Figure 10:** Sample instances generated by GAN.

**Figure 11:** Original insoluble image.

**Figure 12:** Feature plots at different scales.

**Figure 13:** Comparison of different fold cross-validation.

**Figure 14:** Model accuracy comparison under different hidden layers.

**Table 1:** Data distribution tables.

	Total datasets (2250)	Training sets (1800)	Test sets (450)
Low solubility	931	737	194
Medium solubility	668	542	126
High solubility	651	521	130

**Table 2:** Comparison of accuracy on the test set for model cross-validation per fold and with and without cross-validation (%).

Model	Fold-1	Fold-2	Fold-3	Fold-4	With cross-validation	Without cross-validation
GAN-ELM	44.66	45.11	44.00	47.55	64.00	51.66
GAN-ELM-L1	49.55	48.44	53.55	50.44	67.55	58.22
GAN-CNN-ELM	97.66	96.99	97.22	96.33	98.91	97.66

**Table 3:** Model comparison.

Model	Features (number of input features)	Total feature extraction time (unit: s)	Duration of training (unit: s)	Total time (unit: s)	Accuracy (%)
GAN-CNN	—	—	—	5153.56	97.78
GAN-ELM	15360	1250.51	3.96	1254.47	53.78
GAN-ELM-L1	15360	1250.51	3.11	1253.62	59.33
GAN-SVM	15360	1250.51	14.83	1265.34	54.61
GAN-CNN-SVM	15360	1250.51	13.47	1263.98	98.61
CNN-ELM	15360	1085.28	3.41	1088.69	97.97
GAN-CNN-ELM	15360	1250.51	3.44	1253.95	98.77

**Table 4:** Comparison of CNN, CNN-SVM, and CNN-ELM recognition efficiency comparison.

Model	Data size (unit: amplitude)	Identification time (unit: s)	Recognition accuracy (%)
GAN-CNN	450	172.56	94.55
GAN-CNN-SVM	450	54.62	95.89
CNN-ELM	450	39.66	96.33
GAN-CNN-ELM	450	38.28	98.91

## Data Availability

The image data used to support the findings of this study are included within the article.
